# Evaluating the Impact of Community Experience on Purchase Intention in Online Knowledge Community

**DOI:** 10.3389/fpsyg.2022.911594

**Published:** 2022-06-14

**Authors:** Hong Zhao, Qiaohong Shi

**Affiliations:** ^1^International College of Cultural Education, Northeast Agricultural University, Harbin, China; ^2^College of Finance and Economics, Nanchang Institute of Technology, Nanchang, China

**Keywords:** information experience, entertainment experience, sociability experience, brand identity, purchase intention

## Abstract

Community experience has an important influence on the brand building of an online knowledge community. By enhancing the community experience of members, it can promote the building of an online knowledge community and increase users' purchase intention. Although existing research has explored the influence model of community experience, there is a dearth of research regarding the influence of community experience on purchase intention. To this end, this study uses the online knowledge community experience as a theoretical basis to construct a mediating model to examine the behavioral patterns of consumers using the online knowledge communities and to explore in detail the mechanisms of the different dimensions of the community experience on purchase intention. It was found that not only the three dimensions of community experience (i.e., information experience, entertainment experience, and interactive experience) had a significant effect on brand identity, but also brand identity had a significant effect on purchase intention. The study also confirmed that brand identity mediates the relationship between community experience and purchase intention. This study reveals the mediating mechanism of community experience on purchase intention and helps to effectively guide the innovative management practices of the online knowledge community.

## Introduction

In the era of rapid development of 5G technology, cloud computing, and big data, the learning scenario of the online knowledge community is becoming a major measure for companies to attract and retain customers, opening up a new model of a learning experience for users with the support of new technologies (Kaur et al., 2020; Zhao et al., 2021). The innovation of information technology has greatly driven the development of the experience economy, and companies and brands are trying to deepen members' identification with the brand by providing various experiences for online knowledge community members, and bringing more suitable products to different users, so as to increase users' purchase intention (Han and Zhou, 2020; Yuan et al., 2021). Therefore, as a key link to strengthen its own connection with users, the online knowledge community may be another differentiating direction and option for corporate branding (Garay and Morales, 2020). Therefore, research to clarify the internal logic between the value of online knowledge community experience and customers' willingness to purchase can not only enrich academic research but also help companies' practice. User experience can improve the quality of the online knowledge community and the value of the experience in participating in an online knowledge community, and this value, built on brand experience, can contribute to the growth of the online knowledge community (Sun, 2020). Research suggests that as the environment changes, the focus of economic activity is no longer on output, but on consumption in the form of experiences, and consumers focus on the pursuit of sensations and expect to enjoy the cascade of immersive experiences that companies provide (Wang et al., 2021). In this situation, the online knowledge community, which provides users with experiential value, has a growing influence on users' brand identity. Thus, it is clear that the online knowledge community, as a typical virtual brand community, has an important influence on brand building through its members' experience value, which helps the online knowledge community achieve a virtuous cycle between brand building and brand enhancement (Liao et al., 2020a; Deng et al., 2021). Currently, academics have conducted related research on the online knowledge community (Chen et al., 2019; Lin et al., 2019; Yang et al., 2020; Zhao et al., 2021).

First, this research discusses the influence of users' motivation to participate and participation behavior on their brand loyalty. Prior research suggests that consumers participate in communities to search for product-related information or to communicate emotionally (Wang et al., 2020). By providing a place for users to communicate with each other in the form of the online knowledge community, companies can bring more opportunities for suppliers and customers, which is a potential way to increase customer loyalty (Qiao et al., 2021). However, these studies mainly follow the “motivation–behavior–outcome” behavioral model, which helps to provide practical responses to consumer behavior, but ignores the psychological evolutionary stage of “perception–attitude–behavior”, i.e., the influence of individual's psychological perception on behavior and outcomes. As community members' perceptions are formed through their experience of the community, community experience as an antecedent of members' perceptions will have an important impact on the formation of their brand identity and brand use behavior. Therefore, it is necessary to explore the specific components of virtual brand community experience and analyze the specific degree and form of influence of members' experience on brand-related factors (Xiao, 2018; Berni et al., 2020).

Second, our research is based on the content of online knowledge community user activities. The research on online knowledge community experience is still in its infancy, and most of the scholars mainly focus on the perspective of “the content of members' activities in the community” (Ye and Lin, 2021). Li et al. (2021) argued that community value co-creation can achieve user support for the community, and used social network embedding as the independent variable, value co-creation as the dependent variable, self-determination as the mediating variable, and community support as the moderating variable to construct a theoretical model of the mechanism of the effect of social network embedding on virtual community value co-creation, and used structural equation modeling (SEM) to test the influence of relationships among social network embedding, virtual community value co-creation, self-determination, and community support through field research. Huo et al. (2019) concluded that customer participation in spontaneous brand co-creation positively influences firm-initiated brand co-creation; firm-initiated brand co-creation plays a partially mediating role between spontaneous brand co-creation and customer value dimensions. It can be seen that the online knowledge community has become an important platform for interaction between companies and users, and it is important to develop online knowledge community interaction to establish user fitness. In-depth research on the relationship between online knowledge community testing and user fitness is in line with current practice (Liu et al., 2019; Wen et al., 2021). However, researchers have not yet generalized, integrated, and explored the concept of “user community experience in online knowledge community” within the same framework of its specific dimensional components.

Third, some scholars who study the business value of the online knowledge community and the impact of the online knowledge community on brands often use case studies. The lack of research on the composition of the experience dimensions of online knowledge community members makes it difficult to conduct empirical research on the influence of online knowledge community members' psychological perceptions on brand attitudes. For example, in a study examining whether and how perceived interactivity in virtual community influences brand preferences for brand sustainability, Li et al. (2021) tested that values (social, emotional, and informational values) have a positive impact on brand preferences through data collected in online communities. While this study provides reliable and important brand management strategies for the online knowledge community, it does not further explore the impact of individual purchase intentions. Although there are a few empirical studies on the influence of communities on brand-related factors, such as Han and Zhou (2020), which experimentally explored the mechanism of experiential user-generated content on other users' purchase intentions in a social e-commerce community, they did not examine the applicability of different types of values in the community by discussing the “bandwagon” phenomenon from the Little Red Book community. The applicability of different types of values in the community is not examined. If the specific constituent dimensions of the online knowledge community experience and the way and extent to which it influences brand identity can be explored through empirical research to derive a community experience impact model on the brand, then companies can be guided in a targeted manner to establish online knowledge community to better guide users' brand. The study also explores the specific dimensions of the online knowledge community experience and how and to what extent it affects brand identity.

The above-mentioned analysis shows that while previous studies have achieved a series of fruitful results, they also have some shortcomings. First, although scholars have identified experience as a key factor influencing the online knowledge community, they have examined its role more as a single-dimensional concept. Although these findings can reveal the positive significance of community experience, it is difficult to reveal the differentiated impact results of different dimensions of community experience in community activities, which in turn limits the usability of the research findings. Second, previous research has often focused on the impact of user community involvement on community identity or product attitudes, ignoring how and what impact the user community experience has on purchase intentions, when in fact user purchase is what builds the value of a company's brand identity. Finally, it has been pointed out that existing studies often lack the exploration of the mediating variables from community experience to brand identity, which makes the mechanism of the role of online knowledge community zones not easy to be clearly explained. Therefore, this study takes the virtual brand community experience as the theoretical basis, proposes a new model as the theoretical basis for the study, takes users of the Thousand Chat community as the research object, uses structural equation modeling (SEM) to examine the behavior patterns of users using online knowledge community, and explores in detail the influence of different dimensions of community experience on purchase intention. It is hoped that this study will provide a useful reference for the practice of online knowledge community and provide a comprehensive, in-depth, and detailed understanding of the differentiated needs of users, with a view to promoting the promotion of online knowledge community and bringing about greater market synergy.

## Theoretical Foundation and Hypothesis Development

### Online Knowledge Community Experience

The study concluded that the online knowledge community is a typical virtual brand community (Lin et al., 2019; Yang et al., 2020; Zhao et al., 2021). Kozinets (2002) defines a virtual brand community as an “online brand community,” which means that members of a brand community communicate mainly through the Internet, mostly through brand forums, personal homepages, and blogs, to share their brand experiences and attitudes toward brands. Virtual brand communities as a kind of content-generating online communities or forums are social networks initiated by companies, brand followers, or third parties and formed based on digital communication technologies (Liao et al., 2020b). Thus, users can discuss brand knowledge and share brand experiences and feelings in virtual brand communities (Lima et al., 2019). In recent years, domestic and international marketing scholars have focused on the impact of virtual brand communities on the behavior of community members. For example, Wen et al. (2021) proposed a research model on the effect of virtual brand community interactions on customer fit, which introduced mind-flow experience as a mediating variable into the conceptual model and explored the moderating role of remote presence, and validated the research framework through 2 × 2 manipulative scenario experiments and questionnaire data. The results showed that both interpersonal and social-like interactions had a significant positive effect on customer fit, both interpersonal and social-like interactions had a significant positive effect on mind-flow experience, mind-flow experience mediated the interaction between virtual brand communities and customer fit, and remote presence moderated the interaction between social-like interactions and mind-flow experience, i.e., when members of the virtual brand community were engaged in social-like interactions in the virtual brand community, they had a positive effect on customer fit. The higher the level of remote presence perception, the stronger the mind-flow experience. Huo et al. (2019) constructed a hypothetical model of the impact of the type of customer participation in brand co-creation on each dimension of customer value, and Ye and Lin (2021) constructed a model of the drivers of user participation in value co-creation behavior in virtual brand communities.

At present, academic research on online knowledge community experience has achieved certain results, and there are rich discussions and studies on its specific composition dimensions. Summarizing the existing literature, this paper observed that users in online knowledge communities experience their communities in the following three aspects. First is information experience, i.e., users' experience of acquiring or sharing information in an online knowledge community. Flanagin and Metzger (2001) argue that community members tend to use online knowledge communities as a tool to accomplish specific tasks and purposefully collect and process information in virtual communities. Kim et al. (2004) conducted a study on the communities of some Korean tourism companies and found that the satisfaction of users' needs is a key determinant of their online community experience, and the most important of these needs is the access to information. If users feel that they can get valuable information from the community, can exchange valuable information with each other and other members of the community, and are very satisfied with the information provided by the community, then users will be more involved in the online knowledge community and will be further loyal to the company's products. Second, entertainment experience, i.e., the user's relaxed and enjoyable feeling through browsing content in virtual communities, is the most basic and important factor for the online knowledge community, including scenes, content, activities, music, and graphics. Pine and Gilmore (1999) showed that the entertainment experience is a pleasurable and relaxing experience for the user by browsing the content in the virtual community or by perceiving the aesthetics of the community design (e.g., pictures, images, and flash). Third, sociability experience is the experience that users get by communicating with others in the online knowledge community. Leung (2003) argues that the sociability experience is an experience in which members of a virtual community engage in virtual community activities and gain friendship and social support through contact and communication with people who share similar ideas in order to dispel loneliness.

With the support of information technology, the online knowledge community becomes the communication medium between companies and users, so creating a good online knowledge community experience environment can effectively maintain user relationships (Elia et al., 2020). Clearly, community experience has become a powerful tool for companies to win users, as users focus on sensory pursuits and expect companies to provide an immersive environment. Research has found that in an online knowledge community, users' community experience has a positive and significant impact on their brand perceptions, and when users' community experience matches their expectations, they tend to respond positively to marketing activities promoted by the online knowledge community (Zhao et al., 2021). Therefore, enabling users to achieve a good community experience and establish a long-term trust relationship with them will be a key issue for companies to address when branding in the virtual economy. Therefore, this study uses community experience as a theoretical basis to discuss the influence of online knowledge community experience on users' willingness to purchase.

### The Impact of Community Experience on Brand Identity

Research suggests that an important determinant of brand identity and brand equity is the customer experience during the service process (Nambisan and Watt, 2011). With the increasing development of mobile Internet technology and virtual economy, the online knowledge community experience is playing an increasingly important role in modern brand marketing. Community experience is a subjective perception of the benefits (difference between output and input) that people receive from participating in an online knowledge community, which is a response to the external environment (online knowledge community). Brand identity is the subjective cognition of consumers who use past experiences to understand, perceive, and evaluate the information of the brand, which is a kind of individual psychological experience and cognition (Wang et al.'s, 2019). The various types of community experiences that consumers receive in the online knowledge community are the messages that the company wants to convey to its users, and individuals will form a brand identity for the company based on the experiences they receive. Studies on the influence of online knowledge community on users' willingness to purchase new products through group identity and brand identity have found that online knowledge community experiences indirectly influence new product purchase intentions through group identity and brand identity, and that user community experiences are an important influence on group identity and brand identity in the online knowledge community environment. Through this study, it is known that user community experience in an online knowledge community has a positive influence on brand identity (Li et al., 2017). Undoubtedly, in order to better improve the impact of online knowledge community experience on brand identity, the online knowledge community is required to pay attention to various needs of users, actively build and improve the experience value of the community, actively provide various experiences needed by users, and prompt users to spontaneously become brand promoters. Companies are required to provide facilitation conditions in the actual operation of the online knowledge community and actively promote users' online knowledge community and brand identification (Huang and Chen, 2018).

Aswani et al. (2018) suggested that when users achieve a community experience in an online knowledge community, individuals will develop a more positive assessment of this brand identity, such as when companies use the online knowledge community to quickly provide users with the most comprehensive experience based on empowering customers with an effective, quality brand identity. This coincides with Das et al. (2019), who argue that community experiences have a positive effect on users' formation of positive brand identity. Combined with Wang et al.'s (2019) study, which classifies online knowledge community experiences into informational, entertainment, and sociability experiences, it is argued that these three dimensions can positively influence brand identity through users' psychological perceived usefulness and perceived ease of use. It can be inferred that users' brand identification with virtual communities depends on their perceptions of the experiences that online knowledge communities can provide. If an online knowledge community can provide a high level of the community experience for its members, it will not only meet their needs well, but also enhances the influence and attractiveness of the community itself, and makes it easier for the community members to form strong emotional bonds with each other. Therefore, the greater the value of the experience users receive in the online knowledge community context, the better the brand identity of the online knowledge community. Based on the aforementioned arguments, this paper proposes the following hypotheses.

H1a: Information experience is positively associated with brand identity.
H1b: Entertainment experience is positively associated with brand identity.
H1c: Sociability experience is positively associated with brand identity.

### The Influence of Brand Identity on Purchase Intention

Lastovica and Gardner (1979) first defined brand identity as the degree to which consumers are emotionally or psychologically attached to a brand, and based on their study of brand connotations, found that consumers often base their purchase decisions on brand identity. In other words, consumers' brand identity has a decisive influence on their purchase intentions. According to Río et al. (2001), brand identity can be divided into personal identification and social identification, while Šerić et al. (2017) argues that brand identity can be divided into two levels, emotional identification and emotional experience, where emotional identification is the highest level of brand equity and reflects a completely harmonious relationship between the brand and the consumer. According to this study, brand identity is the degree of overlap between consumers' perceived self-concept and brand concept. Enterprises can provide a platform for consumers or potential consumers to communicate with each other through the establishment of an online knowledge community, and this horizontal communication between consumers can strengthen each other's identity with the brand.

Users' experiences with an online knowledge community often begin with the operability of that community, and the simplicity and ease of operation enhance users' positive perceptions of the functionality of the online knowledge community. Bagozzi and Dholakia (2006) argue that brand communities influence consumer brand perception and brand behavior. This study found empirically that virtual community brand identity can promote consumer brand purchase behavior. Based on Gong et al.'s (2021) explanation of how brand positioning strategies positively influence consumer responses, it can be inferred that individual brand identity contributes significantly to consumers' purchase intentions and recommendation intentions. The prerequisite for consumers to identify with the online knowledge community they belong to is sufficient knowledge of the community, and users tend to identify with the online knowledge communities that can enhance their self-worth (social status, social image) and consequently develop a sense of belonging to the community. In this case, users have a better perception of their online knowledge community and differentiate it from other communities, and are more emotionally invested in their online knowledge community, which helps them to strengthen their self-definition and self-image. Accordingly, users will differentiate the online knowledge community they identify with from other communities and resist competing brands, such as refusing to join other communities and refusing to buy other brands' products. In the same way, it can be inferred that the brand identity of online knowledge community has a positive impact on purchase intentions. As such, this paper expects that brand identity will drive users to attain higher purchase intention.

H2: Brand identity is positively associated with purchase intention.

### Mediating Role of Brand Identity

In his study, Bagozzi and Dholakia (2002) pointed out that an individual's identification with an online knowledge community is a state of mind in which the individual identifies himself or herself with other members of the online knowledge community and sees himself or herself as part of that online knowledge community. The findings of Zhang (2021) and Zhang (2022) similarly support the idea that community experience has an impact on brand identity, as they suggest that individuals identify with an online knowledge community based on community benefits, i.e., members perceive that the community provides their desired value. The findings of Wang et al. (2020) and Li et al. (2021) also provide support for the influence of community experience on brand identity. The level of brand identity depends on the community members' perceptions of the various experiences offered by the online knowledge community. An online knowledge community that provides a high level of service to its members not only satisfies their corresponding needs well, but also enhances the influence and attractiveness of the community itself and makes it easy for strong emotional bonds to be formed among community members.

Based on the above-mentioned analysis, this paper can find that the community experience (information experience, entertainment experience, and sociability experience) of the online knowledge community has a positive impact on the brand identity. The community experience (information experience, entertainment experience, and sociability experience) provided by the online knowledge community can meet the different needs of the community members and continuously enhance the community members' identification with the online knowledge community, i.e., generate brand identity.

Schau and Muniz (2002) argue that the online knowledge communities influence consumers' brand perceptions and brand behavior, and Bagozzi and Dholakia (2006) find empirically that brand community identification promotes consumers' brand purchase behavior. Ren et al. (2007) categorized community identity into individual and community identity and confirmed through empirical studies that individual identity and social identity have a significant contribution to consumers' purchase intention and recommendation intention. Users tend to identify with an online knowledge community that enhances their self-worth (social status and social image) and thus develop a sense of belonging to that community. When users identify with an online knowledge community, they are more likely to purchase the brand again, which is also necessary to maintain a sticky relationship with the online knowledge community. Based on the above-mentioned analysis, it can be found that the brand identity of online knowledge community members has a positive influence on the purchase intention of community members. After users identify with an online knowledge community, they are more likely to purchase the brand again.

In summary, since user community experiences (information experience, entertainment experience, and sociability experience) in an online knowledge community have a positive and significant effect on brand identity, brand identity has a positive and significant effect on purchase intention. Therefore, brand identity mediates the relationship between community experience (information experience, entertainment experience, and sociability experience) and purchase intention. In other words, brand identity mediates the relationship between online knowledge community experience (information experience, entertainment experience, and sociability experience) and purchase intention of community members. Based on the above-mentioned comprehensive analysis, this paper proposes the following hypotheses:

H3a: Brand identity plays a mediating role between users' information experience and purchase intention.
H3b: Brand identity plays a mediating role between users' entertainment experience and purchase intention.
H3c: Brand identity plays a mediating role between users' sociability experience and purchase intention.

In summary, this study proposes a research model as shown in Figure 1.

**Figure 1:** Theoretical model.

## Methods

### Participants and Procedure

This study chooses the Thousand Chat community as the research background. Thousand Chat community was established by Tencent in 2011 and is a leading online knowledge community in China. The elites in various fields share their expertise and experience live every day and interact in real time. Currently, the Thousand Chat community has gathered a large number of users who like online knowledge products. In this paper, a questionnaire survey was conducted among Thousand Chat community members to test the hypothesis of this paper. Specifically, the questionnaire for this study was designed in Questionnaire Star, and after the web link was generated, Thousand Chat community members were invited to fill out the questionnaire, and all respondents were informed that “all information obtained from the survey is for academic research only,” “only comprehensive statistical processing of the questionnaire data will be done, no case study will be done. There are no right or wrong answers,” “the questionnaire is filled in anonymously,” and “your information will be kept absolutely confidential.” To encourage users to participate, respondents can get 5 RMB after completing the survey. The survey period was from September 2021 to January 2022, and after 5 months of questionnaire collection, 612 questionnaires were received. After eliminating non-members of the Thousand Chat community or some other invalid questionnaires, 486 valid questionnaires were left, with an efficiency rate of 79.41%. The criteria for a valid questionnaire were that the respondent was a member of the Thousand Chat community and that the respondent was 18 years old or older. In the sample, the gender ratio was 49.8%:50.2%, and the age distribution was 7 people under 19 years, 203 people between 20 and 29 years, 206 people between 30 and 39 years, 52 people between 40 and 49 years, and 18 people over 50 years. Regarding the distribution of education level, 62 people have a college education, 381 people have a bachelor's degree, and 43 people have a master's degree or above. Regarding the average monthly consumption level, 30 people had a monthly consumption of RMB 2,000 or less, 71 people had a monthly consumption of RMB 2,000–3,999, 116 people had a monthly consumption of RMB 4,000–5,999, and 269 people had a monthly consumption of RMB 6,000 or more. The details are summarized in Table 1.

**Table 1:** Descriptive statistical analysis.

**Variables**	**Item**	**Frequency**	**%**	**Cumulative %**
Gender	Male	242	49.8	49.8
	Female	244	50.2	100.0
Age (year)	19 or less	7	1.4	1.4
	20–29	203	41.8	43.2
	30–39	206	42.4	85.6
	40–49	52	10.7	96.3
	50 or above	18	3.7	100.0
Marriage	Married	323	66.5	66.5
	Unmarried	162	33.3	99.8
	Divorce	1	0.2	100.0
EE	Student	57	11.7	11.7
	Freelance	33	6.8	18.5
	Executive in private enterprise	161	33.1	51.6
	Civil servant	210	43.2	94.9
	Clerk in state owned enterprise	20	4.1	99.0
	Executive in private enterprise	5	1.0	100.0
Education	College and blow	62	12.8	12.8
	Undergraduate	381	78.4	91.2
	Master's degree and above	43	8.8	100.0
Consumption (RMB)	Below 2,000	30	6.2	6.2
	2,000–3,999	71	14.6	20.8
	4,000–5,999	116	23.9	44.7
	6,000 or more	269	55.3	100.0
Continuous use time (year)	<1	70	14.4	14.4
	1–2	207	42.6	57.0
	Over 3	209	43.0	100.0

### Measures

This section will describe the measurement tools used in this study, using the Likert scale (1 = Strongly disagree, 7 = Strongly agree). The variable measurements and their sources are as follows.

To measure the information experience, this paper used the three-item scale from Nambisan and Watt (2011) and Wang et al. (2019) that was specifically developed to measure value experience caused by participants' perceived usefulness of information during community activities. Sample items include “I can provide the community with information that others need” and “I can find some solutions to problems in the community.”

To measure the entertainment experience/pleasant experience associated with the participant's participation in community activities or interaction with community members, this paper used the entertainment experience scale developed by Nambisan and Watt (2011). This paper used three items based on the relevance of the recreational content to the community setting. Participants indicated that they had a pleasant experience when participating in community activities or interacting with community members, and sample items for learning include “The content of the community is interesting to me” and “The community can help me relieve the pressure.”

To measure the sociability experience, similar to Yang et al.'s (2021) study, this paper used three items from the Nambisan and Watt (2011) measure and the Wang et al. (2019) measure. Participants indicate the experiences they have gained in the community through interaction with other members, and sample items include “I can get positive feedback from community members,” “The community allows me to better communicate with other members,” and “The interaction in the community impresses me deeply.”

To measure the brand identity, this paper used the three-item scale from Sasmita and Suki (2015), which was developed specifically to reflect the symbolic meanings and self-expressed identities embodied by users in the online knowledge community. Participants indicated their psychological state of being similar to other members of the online knowledge community and seeing themselves as part of that online knowledge community, and sample items include “This particular brand is well established” and “This particular brand has a differentiated image in comparison with the other brand”.

To measure the purchase intention, this paper used the entertainment experience scale developed by Pavlou (2003) and Lin et al. (2011). The scale that was used was made up of four items that measured the intention, the susceptibility to purchase, and the probability of purchase. Sample items include “Given the chance, I intend to purchase from [name of the company]” and “Given the chance, I predict that I should purchase from [name of the company] in the future.”

### Research Methods

This study used structural equation modeling to test and analyze the hypothesized relationships and structural models (SEM) in the study model. Structural equation modeling has the unique advantage of meticulously processing the data to both predict the remaining estimated residuals and analyze measurement error, thus making SEM's definition of latent variables more consistent with the psychometric structure. Therefore, this study applied the Amos 24.0 to analyze the collected data for structural equation modeling.

## Data Analysis and Results

### Measurement Model Analysis

This study evaluates and revises the measurement model of confirmatory factor analysis (CFA) according to the approach of Anderson and Sullivan (1993). That is, CFA should report factor loading, Cronbach's alpha, composite reliability (CR), and average variance extracted (AVE) for all variables, and only after these metrics pass the test, structural model evaluation can be performed (Kline, 2011). Fornell and Lacker (1981), Nunnally and Bernstein (1994), and Hair et al. (2017) clearly stated that when the factor loading is >0.50, Cronbach's alpha is >0.70, the CR is >0.60, and the AVE is >0.50, then the measurement model has good convergent validity.

The indicators of interest for the CFA are reported in Table 2. In this study, factor loadings of all dimensions are between 0.607 and 0.899, Cronbach's alpha is between 0.738 and 0.845, CR is between 0.756 and 0.844, and AVE is between 0.512 and 0.578. Thus, the results of the factor loading, Cronbach's alpha, CR, and AVE meet the criteria of Fornell and Lacker (1981), Nunnally and Bernstein (1994), and Hair et al. (2017). Therefore, the results of the CFA analysis indicate good convergence validity for all the constructs.

**Table 2:** Confirmatory factor analysis.

**Construct**	**Item**	**Factor loadings**	**Cronbach's alpha**	**CR**	**AVE**
Information experience (IE)	IE1	0.711	0.775	0.778	0.539
	IE2	0.714			
	IE3	0.775			
Entertainment experience (EE)	EE1	0.679	0.777	0.797	0.571
	EE2	0.899			
	EE3	0.667			
Sociability experience (SE)	SE1	0.607	0.738	0.756	0.512
	SE2	0.698			
	SE3	0.825			
Brand identity (BI)	BI1	0.661	0.779	0.781	0.545
	BI2	0.778			
	BI3	0.770			
Purchase intention (PI)	PI1	0.839	0.845	0.844	0.578
	PI2	0.836			
	PI3	0.715			
	PI4	0.632			

Table 3 reports the discriminant validity for the measurement model, where the square roots of the AVE are reproduced on the diagonal. Discriminant validity is the extent to which the measure is not a reflection of some other variables. It is indicated by low correlations between the measure of interest and the measures of other constructs. This paper has examined discriminant validity using Fornell and Lacker's (1981) recommendation that the square root of the average variance extracted for each construct should be higher than the correlations between it and all other constructs. Table 3 shows that the squared root of the average variance extracted for each construct is greater than the correlations between the constructs and all other constructs. The results support Fornell and Lacker (1981)'s requirement of discriminant validity.

**Table 3:** Discriminant validity for the measurement model.

**Variables**	**Mean**	**SD**	**AVE**	**1**	**2**	**3**	**4**	**5**
1. Information experience (IE)	5.221	1.019	0.539	0.734				
2. Entertainment experience (EE)	4.314	1.175	0.571	0.427	0.756			
3. Sociability experience (SE)	5.048	1.018	0.512	0.567	0.432	**0.716**		
4. Brand identity (BI)	5.396	1.067	0.545	0.584	0.447	0.542	**0.738**	
5. Purchase intention (PI)	4.916	1.196	0.578	0.515	0.334	0.628	0.560	**0.760**

*The diagonal value is the square root of AVE*.

### Structural Model Analysis

In this study, model fit was analyzed according to the recommendations of Jackson et al. (2009). The results found MLχ^2^ = 118.504, DF = 97, 1 < Normed Chi-sqr (χ^2^/DF) = 1.222 < 3, RMSEA = 0.021 < 0.08, SRMR = 0.026 < 0.08, TLI (NNFI) = 0.992 > 0.9, CFI = 0.993 > 0.9, GFI = 0.965 > 0.9, and AGFI = 0.942 > 0.9. This indicates that the structural model of this study has a good fit (Bollen and Stine, 1992). The path coefficients are shown in Table 4. Information experience (IE) (b = 0.366, *p*-value < 0.001), entertainment experience (EE) (b = 0.139, *p* < 0.01), and sociability experience (SE) (b = 0.404, *p*-value < 0.001) are positively associated with brand identity (BI). Therefore, H1a, H1b, and H1c are established. Brand identity (BI) (b = 0.888, *p*-value < 0.001) is positively associated with purchase intention (PI). Therefore, H2 is established.

**Table 4:** Regression coefficient.

	**Unstd**	**S.E**.	**Unstd./S.E**.	**Std**.	***p*-value**
H1a: IE->BI	0.366	0.071	5.171	0.361	***
H1b: EE->BI	0.139	0.047	2.987	0.163	**
H1c: SE->BI	0.404	0.084	4.786	0.342	***
H2: BI->PI	0.888	0.086	10.280	0.632	***

** *p-value < 0.01,*

*** *p-value < 0.001.*

*IE, Information experience; EE, Entertainment experience; SE, Sociability experience; BI, Brand identity; PI, Purchase intention*.

The results of the mediating effect analysis are shown in Table 5. In this study, structural equation modeling was used to analyze the mediating effect, and the standard error of the mediating effect was first estimated using the Bootstrap estimation technique, and then the significant level of the mediating effect was further calculated. According to Hayes (2009), a mediating effect is indicated if “0” does not include the 95% confidence interval of Bias-corrected, the z-value is >1.96, and the *p*-value is <0.05. Specifically, the total effect of information experience (IE) on purchase intention (PI) is 0.325. At the 95% confidence level, “0” does not include the Bias-corrected 95% confidence interval range, the z-value is >1.96, and the *p*-value is <0.05. Therefore, a total effect exists. The indirect effect is 0.325, “0” does not include the Bias-corrected 95% confidence interval range, the z-value is >1.96, and the *p*-value is <0.05. Therefore, there is an indirect effect. In the same analytical approach, the results of the study show that hypotheses H3b and H3c are significant.

**Table 5:** The analysis of mediating effect.

**Effect**	**Path coefficient (β)**	**Bootstrap 1,000 times**			
		**Bias-corrected 95%**		**Percentile 95%**	
		**Lower bound**	**Upper bound**	**Lower bound**	**Upper bound**
Total effect: IE → PI	0.325	0.110	0.585	0.113	0.585
Indirect effect: IE → BI → PI	0.325	0.110	0.585	0.113	0.585
Total effect: EE → PI	0.124	0.031	0.220	0.029	0.217
Indirect effect: EE → BI → PI	0.124	0.031	0.220	0.029	0.217
Total effect: SE → PI	0.359	0.149	0.648	0.130	0.634
Indirect effect: SE → BI → PI	0.359	0.149	0.648	0.130	0.634

*IE, Information experience; EE, Entertainment experience; SE, Sociability experience; BI, Brand identity; PI, Purchase intention*.

## Research Results and Discussion

### Findings and Discussion

First, the findings suggest that community experience has a significant and positive effect on brand identity. The online knowledge community experience helps to enhance the perception of members' brand identity, which is consistent with the existing studies. The reason for this is that users of an online knowledge community can satisfy their needs for relevant information through community experience, recognize the role of the community in improving the efficiency of searching for brand information, easily get the information they need, and increase their identification with the virtual community. The community experience can help members understand product recommendation information, share others' experiences and product reviews, get reliable solutions to some problems, and make friends and form social circles, thus enhancing members' brand identity.

Second, the findings suggest that brand identity has a significant and positive effect on purchase intention. In an online knowledge community, user brand identity helps to enhance members' purchase intentions, which is consistent with existing research. The reason for this may be inferred from the fact that users in online knowledge communities are more inclined to believe in their own brand identity in online knowledge community, while the physical attributes of the communities themselves, such as simplicity of operation and timeliness of communication, are relatively less likely to attract members' attention. Therefore, a more effective way to increase purchase intention is to directly enhance the identification of online knowledge community members in the community, such as initiating multiple discussion topics, opening various forums related to brand information, and creating a composite communication platform to enhance the effectiveness of brand identification in online knowledge community.

Third, the findings suggest that the mediating role of brand identity is validated. In online knowledge community, brand identity mediates the relationship between community experience and purchase intentions, which is consistent with existing research. The physical attributes of online knowledge community do not allow members to associate their personality characteristics with the values and behavioral concepts represented by the brand, but only through repeated communication, interaction, and identification in the online knowledge community can brand identity be generated. In short, in the online knowledge community environment, the key to brand identity for members lies in the community experience, and the generation of community experience depends on the actual experience of users in the community and also on the physical attributes of the community itself.

### Theoretical Contributions

First, this paper explores the influence and role of online knowledge community on users' purchase intention based on a community experience perspective, and confirms the influence mechanism of online knowledge community experience on product purchase intention, which enriches the theoretical study of online knowledge community on brand product promotion and proves that user community experience in online knowledge community is an important influencing factor for brand promotion. While previous related studies focused on the influence of user involvement, interaction level, and innovation atmosphere of online knowledge community on brand promotion, this paper confirms that user community experience is also an important driver of brand promotion.

Second, this paper classifies community experience into information experience, entertainment experience, and sociability experience, and verifies the mechanism by which different content experiences of online knowledge community users affect users' willingness to purchase products. This not only enriches the theoretical research on online knowledge community experience and brand promotion, but also expands the use of online knowledge community experience and proves that the segmentation dimension of community experience is an important facilitator of product promotion. While previous studies on the perceived value of the online knowledge community focused on the impact of perceived value on user satisfaction, brand commitment, and brand loyalty, this study confirms that community experience is also an outcome variable of brand identity and ultimately influences purchase intention.

Third, the empirical results of this paper confirm that user community experience is an important influencing factor of brand identity in the online knowledge community environment. While previous studies on the factors influencing virtual brand identity have mainly considered satisfaction, interaction, and brand relationship quality, the findings of this study broaden the scope of this study. Moreover, the mechanism and three paths by which online knowledge community experience influences brand promotion have more specific and practical implications for corporate marketing practices.

### Practical Implications

First, managers should start to improve the user experience of the online knowledge community, and actively guide users' brand identification tendency by deepening the experience and improving the perceived usefulness and ease of use. The online knowledge community should pay attention to the various experience needs of users and set up a special service team to investigate the experience needs of users, and on this basis, actively build and improve the various functions of the community and actively provide various experiences that users need, such as brand and product-related knowledge, various discount activities, convenient and smooth sociability experiences among community members, and various activities and games that can delight users. Users get information, and financial, social, entertainment, and other value satisfaction in the online knowledge community, and will become brand promoters spontaneously.

Second, in the actual operation of online knowledge community, since group identification and brand identification have a positive effect on brand promotion, companies should provide facilities to actively promote users' identification with the online knowledge community and brands. Companies need to pay special attention to the fact that group identity does not directly influence users' willingness to buy new products, but positively influences their willingness to buy through brand identity. This means that while it is important to build group identity in an online knowledge community (i.e., to get users to identify with the online knowledge community), it is not enough to get users to identify with the group in order to achieve the purpose of brand promotion in online knowledge community, and only in this way can the ultimate purpose of brand promotion be realized.

Third, online knowledge community managers need to filter the information effectively so that the community members can find the desired experience in a targeted manner, and delete the false experiences that affect the development of the community in order to ensure the usefulness, reliability, and timeliness of the community information. The community design needs to strive to enhance the interaction motivation of the brand community members through various incentives. For instance, in promoting the online knowledge community, this paper should focus on improving the functionality and convenience of the community and continuously improve the functions of text, links, audio and video, and photo editing, so as to achieve the corresponding improvement in brand identity.

### Research Limitations and Future Research Directions

First, the choice of external control variables is relatively limited. In addition to community experience, there are several factors, such as condition, that can influence member brand identification and thus purchase intentions. However, given that the main purpose of this paper is to study the influence of individual community experience on purchase intention, other factors were not included in the study. Future research could consider adding the influence of other factors, such as environmental characteristics, community characteristics, etc.

Second, this study used questionnaires to empirically test the research hypotheses, and subsequent studies may consider using experimental methods to verify the mechanism of the perceived value of the online knowledge community on users' willingness to purchase new products, so that the many benefits of both methods can be taken into account in the research process.

Third, although the theoretical model used in this study is based on a solid theoretical foundation, the survey method used is a cross-sectional survey method, and the relationship between variables obtained through this cross-sectional research design should be interpreted more as a correlation than a causal relationship. Future studies can consider adding longitudinal surveys, which can test the applicability of the model more comprehensively and thus better explain the relationships among variables.

## Data Availability Statement

The original contributions presented in the study are included in the article/supplementary material, further inquiries can be directed to the corresponding author.

## Ethics Statement

Informed consent was obtained from all subjects involved in the study.

## Author Contributions

HZ: conceptualization and writing original draft. QS: formal analysis and investigation. HZ and QS: writing, reviewing, and editing. All authors have read and agreed to the published version of the manuscript.

## Conflict of Interest

The authors declare that the research was conducted in the absence of any commercial or financial relationships that could be construed as a potential conflict of interest.

## Publisher's Note

All claims expressed in this article are solely those of the authors and do not necessarily represent those of their affiliated organizations, or those of the publisher, the editors and the reviewers. Any product that may be evaluated in this article, or claim that may be made by its manufacturer, is not guaranteed or endorsed by the publisher.
